# CCL3 Promotes Proliferation of Colorectal Cancer Related with TRAF6/NF-*κ*B Molecular Pathway

**DOI:** 10.1155/2022/2387192

**Published:** 2022-07-12

**Authors:** Xiaoqiang Ma, Jinda Su, Shaohui Zhao, Yaqin He, Shuzhen Li, Xiaoliang Yang, Sifan Zhai, Shikuo Rong, Xin Zhang, Guangxian Xu, Xiaoliang Xie

**Affiliations:** ^1^Department of Colorectal Surgery, General Hospital of Ningxia Medical University, Yinchuan 750003, China; ^2^College of Clinical Medicine, Ningxia Medical University, Yinchuan 750004, China; ^3^Surgical Department, General Hospital of Ningxia Medical University, Yinchuan 750003, China; ^4^Operating Room, General Hospital of Ningxia Medical University, Yinchuan 750003, China; ^5^Surgical Department, Lingwu Traditional Chinese Medicine Hospital, Yinchuan 750499, China; ^6^Department of Colorectal and Anal Surgery, First Affiliated Hospital of Zhengzhou University, Zhengzhou 450052, China; ^7^Department of General Surgery, Chengdu Second People's Hospital, Chengdu 610021, China; ^8^Institute of Clinical Laboratory Medicine, Guangdong Provincial Key Laboratory of Medical Molecular Diagnostics, Guangdong Medical University, School of Medical Technology, Dongguan 523000, China

## Abstract

Chemokine C-C motif chemokine ligand 3 (CCL3) plays an important role in the invasion and metastasis of malignant tumors. For developing new therapeutic targets and antitumor drugs, the effect of chemokine CCL3 and the related cytokine network on colorectal cancer should be investigated. This study used cell, tissue, and animal experiments to prove that CCL3 is highly expressed in colorectal cancer and confirmed that CCL3 can promote the proliferation of cancer cells, and its expression is closely related to TRAF6/NF-*κ*B molecular pathway. In addition, protein chip technology was used to examine colorectal cancer tissue samples and identify the key factors of chemokine CCL3 and the toll-like receptors/nuclear factor-*κ*B (TLR/NF-*κ*B) pathway in cancer and metastatic lymph nodes. Furthermore, the lentiviral vector technology was employed for transfection to construct interference and overexpression cell lines. The experimental results reveal the mechanism of CCL3 and TNF receptor-associated factor 6 (TRAF6)/NF-*κ*B pathway-related factors and their effects on the proliferation of colon cancer cells. Finally, the expression and significance of CCL3 in colorectal cancer tissues and its correlation with clinical pathology were studied by immunohistochemistry. Also, the results confirmed that CCL3 and C-C motif chemokine receptor 5 (CCR5) were expressed in adjacent tissues, colorectal cancer tissues, and metastatic cancer. The expression level was correlated with the clinical stage and nerve invasion. The expression of chemokine CCL3 and receptor CCR5 was positively correlated with the expression of TRAF6 and NF-*κ*B and could promote the proliferation, invasion, and migration of colorectal cancer cells through TRAF6 and NF-*κ*B.

## 1. Introduction

According to the data from the International Cancer Research Center of the World Health Organization, in 2020, the number of new cases of colorectal cancer worldwide reached approximately 1.9 million. The incidence and mortality associated with colorectal cancer (approximately 935,000 deaths) rank third and second, respectively, among malignant tumors [1]. Although colorectal cancer can be cured by surgical resection, various factors result in a low rate of early diagnosis, high recurrence and metastasis rates, and poor prognosis, thereby posing great threat to human health [2]. Hence, controlling the metastasis and recurrence of colorectal cancer is a difficult challenge. Chemokines are a class of cytokines that can cause cells to undergo chemotactic movement, and their main role in the body is in chemotactic cell migration. They are widely expressed in various tissues and cells of the body, and their receptors are mainly expressed in white blood cells, mediating the directional migration of white blood cells to play a biological role. In addition, they can also be used as a surface marker of immune cells as they are closely related to cellular immune responses. Tumor cells can also express chemokines and receptors. They can use the “navigation effect” of chemokines, which is closely related to the targeted organ metastasis of tumors [3–5]. CCL3, one of the components of the chemokinep CC ligand family was also termed as MIP (macrophage inflammatory protein). It can be expressed on the surface of macrophages, lymphocytes, epithelial cells, and other cells. It mediates the secretion of cytokines by immune cells and promotes the aggregation and migration of a variety of cells. C-C motif chemokine receptor 1 (CCR1) and CCR5 are the receptors of CCL3. Recent studies have found that CCL3 plays a role in the invasion and metastasis of malignant tumors. A previous study reported that upregulation of CCL3 expression can promote the invasion and migration of lung cancer A549 cells [6]. Silva et al. [7] found that in C57BL/6 (wild type) mice with chemically induced oral squamous cell carcinoma, the expression of CCL3 and CCR5 increased. Of note, knockout of the CCL3 gene retarded tumor cell proliferation. The above studies indicated that the secretion of CCL3 promotes the development of malignant tumors. Studies have demonstrated that liver cancer cell lines produce higher levels of CCL3 than normal cells, which stimulates these cells to produce pseudopodia and migrate *in vitro* [7]. A study using a kidney malignant tumor model found that knockout of the CCL3 and CCR5 genes in mice can reduce the incidence of tumor metastasis [8]. CCL3 is highly expressed in a variety of cancers, but its expression in colorectal cancer has rarely been investigated.

One of the receptors of CCL3 and CCR5 has been studied in depth as an important co-receptor for human immunodeficiency virus type 1 (HIV-1) during invasion of the human body. At present, maraviroc, a targeted CCR5 inhibitor, has been used in the treatment of patients with clinical HIV. However, CCR5 functions as a co-receptor for chemotactic immune cells to mediate HIV invasion of CD4 + T cells [9, 10] and participates in the development of malignant tumors. Nevertheless, in the field of cancer treatment, there is limited evidence regarding the role of CCR5 as a specific marker of certain tumors. A previous study reported that binding of a ligand by CCR5 can activate the GTPase-activating protein, which in turn activates protein kinase C (PKC). This process results in the activation of downstream transcription-related signaling pathways, the p65 subunit of nuclear factor-*κ*B (NF-*κ*B), and the phosphatidylinositol-3-kinase (PI3K) signaling pathway in a secondary cascade [11]. TNF receptor-associated factor 6 (TRAF6) can directly or indirectly bind to members of the TNF receptor superfamily [12], through the activation of the transcription factor PI3K/AKT and activator protein-1 (AP-1) pathway. Therefore, the expression of important factors related to the CCL3–CCR5 axis and TRAF6/NF-*κ*B pathway in colorectal cancer warrants further investigation.

In this study, protein array was used to screen 38 chemokines from 16 tissue samples from colorectal cancer patients initially. After screening, CCL3, which is highly expressed in colorectal cancer tissues, was selected as the target factor. The cancer tissue samples of patients were selected for further verification of expression at the tissue level using immunohistochemical experiments. The correlation between CCL3–CCR5 expression and clinical indicators was further analyzed based on the characteristics of the clinical data of patients with colorectal cancer. To verify the expression of CCL3 in colon cancer and its cancer-promoting effects in cells and animal experiments, CCL3 interference and construction of an overexpression lentiviral vector were performed. Besides, a preliminary study on the interaction between the target factor CCL3 and the differential pathway-related factors (TRAF6, NF-*κ*B, and PI3K) in colon cancer cells was conducted.

## 2. Related Work

The intrinsic properties of tumor cells and the surrounding microenvironment play a vital role in the development and metastasis of tumors. The key steps in their progression and metastasis include proliferation, angiogenesis, invasion, and remote metastasis of tumor cells. All these steps are regulated by chemokines [13].

Structurally, chemokines are divided into three sub-families (CXC, CC, and CX3C). In view of the miniaturization, integration, and high-throughput characteristics of protein array technology, we used protein array for chemokine expression detection and pathway screening in colorectal cancer and adenoma sequence tissues. The subsequent western blotting and immunohistochemical analysis results revealed that the key factors of the target pathways screened were highly expressed in different degrees in colorectal cancer tissues. Although individual chemokines did not match the screening results in the later verification process, protein array technology exhibits certain accuracy in the screening of differential proteins in colorectal cancer tissues. Hence, it can be used for large-scale screening of tumor differential factors and markers.

Studies have used protein antibody arrays to screen colorectal cancer and paracancerous tissue samples. These investigations examined the chemokine CCL5 as a candidate gene and confirmed that it is highly expressed in colorectal cancer [14]. In the present study, we confirmed that CCL3 is highly expressed in colorectal cancer tissues. In addition, Da [15] reported that CCL3 and CCR5 showed high expression in oral squamous cell carcinoma, while normal oral epithelial cells also expressed CCL3. This result is consistent with our findings in colorectal cancer tissues, suggesting that CCL3 is ubiquitous and lowly expressed in human normal epithelial cells. In cells undergoing inflammatory hyperplasia or even cancerous transformation, CCL3 exhibits a trend toward high expression. In normal epithelium and knot tissues, there is a balance between the expression of chemokines and chemokine receptors. Once a certain pathogenic factor disrupts this balance, the cascade reaction caused by the imbalance of homeostasis can lead to malignant consequences [16]. In this study, we confirmed that CCL3 and CCR5 are secreted by macrophages and lymphocytes, and expressed in low levels in normal colonic epithelial cells. Nevertheless, their expression was more obvious in cancer tissues.

CCR5 is expressed in numerous types of cancer and plays an important role in the occurrence and development of a variety of tumors [17]. Furthermore, studies found that malignant tumors can also overexpress CCR5 and accelerate their malignant biological behavior [18–20]. In the tumor microenvironment, in addition to tumor cells, there are lymphocytes, monocytes, fibroblasts, mesenchymal cells, etc. Studies have found that CCR5 is expressed in the above cells [21, 22]. Moreover, the expression of CCR5 in colon cancer tissues is positively correlated with disease aggressiveness and metastatic lymph nodes [23]. Immunohistochemistry experiments combined with correlation analysis of clinical data have found that the expression of CCL3 and CCR5 is correlated with the clinical TNM staging. Of note, the expression of CCR5 is also related to nerve invasion. This phenomenon suggests that CCR5 may be an important factor in the development of certain malignant tumors.

TRAF6 is a key factor that depends on the MyD88 for the toll-like receptors (TLR) pathway. TRAF6 is expressed and distributed in a variety of malignant tumor tissues, including colorectal cancer tissues [24]. In this study, we confirmed that TRAF6 is highly expressed in colorectal cancer tissues. The present finding provides a foundation for further research on pathways. TRAF6 can activate NF-*κ*B in the nucleus through the classical pathway or the alternative pathway and produce biological effects to participate in the process of inflammation and tumor invasion and metastasis [25]. This experiment confirmed that NF-*κ*B and PI3K are both present and highly expressed in colorectal cancer tissues. These findings also laid the foundation for further research on the relationship between the TRAF6/NF-*κ*B pathway and regulatory function of chemokines at the cellular level in the later stage of the disease.

Chemokines are an important part of the tumor microenvironment. In the process of malignant transformation of epithelial cells, various components of the tumor microenvironment are abnormally expressed and secreted through a series of pro-inflammatory molecules, including chemokines, cytokines, and a large number of intracellular signal molecules (such as upstream kinases and transcription factors). This process leads to the formation of an inflammatory state within the tumor, thereby promoting the development of tumors. There is a dynamic relationship between tumor cells and stroma, which promotes the initiation of malignant epithelial cells, leading to tumor immune escape, growth, and metastasis.

NF-*κ*B can regulate a variety of genes in cells to promote inflammatory proliferation, increase metastasis, and inhibit cell apoptosis [26]. Studies have shown that during the progression of the colorectal adenoma-carcinoma sequence, NF-*κ*B promotes the progression of colorectal cancer by inhibiting apoptosis [27]. In addition, it was found that NF-*κ*B can mediate the resistance to TNF-*β*-induced apoptosis in the treatment of colon cancer [28]. As shown in animal experiments, inhibiting the activation of NF-*κ*B prevents the peritoneal metastasis of colon cancer [29]. Activation of NF-*κ*B can promote the expression of matrix metalloproteinases (MMP) and metastasis of colon cancer [30, 31]. Studies have shown that silencing NF-*κ*B can significantly reduce the transformation of inflammatory bowel disease to colon cancer and initiate apoptosis [32]. In our initial experimental design, inflammatory diseases were excluded. However, according to the results, NF-*κ*B remains highly expressed in colorectal cancer tissues, metastatic tissues, colon cancer cell lines, and metastatic cell lines. These findings indicate that this factor is not altered by the occurrence of inflammation in its regulatory network. This study confirmed a positive correlation between the expression of chemokine CCL3 and NF-*κ*B, alterations in the secretion of CCL3, feedback inhibition, and promotion of the expression of NF-*κ*B, which also confirms the existence of a network of interactions.

TRAF6 can activate NF-*κ*B through the activation of cytokine MyD88, CD4, and AP-1 pathways, thereby causing biological effects [33]. TRAF6 and NF-*κ*B interact with each other [34]. Chen et al. [35] found that siRNA blocks the ubiquitination of TRAF6 and activates the inflammatory pathway involved in NF-*κ*B. Therefore, TRAF6 and the NF-*κ*B inflammatory pathway are closely related. This also verified the results regarding the differential pathways screened by the protein array in the second part of this investigation. In this study, we found that interference and overexpression of CCL3 in HT29 and HCT116 cells exerted a positive effect on TRAF6. Combined with the first part of the experiment, there was a positive correlation between the expression of TRAF6 and CCR5 after stimulation of NCM460 cells with bacteroides fragilis toxin-1 (BFT-1). Although the expression of CCL3 was initially decreased, it was subsequently increased. This observation may be related to the dose of the toxin and the stress response of cells to toxic substances. In general, the CCL3–CCR5 axis has an interactive regulatory effect on TRAF6/NF-*κ*B.

Chen et al. [36] conducted studies on cholangiocarcinoma cell lines. They found that stimulation of cells with PI3K inhibitors promoted the apoptosis of cholangiocarcinoma cells; these results were also verified in mouse models of cholangiocarcinoma. Another study reported that in the process of treating bladder cancer and acute lymphoblastic leukemia, activation of the PI3K/AKT signaling pathway can inhibit cell apoptosis and promote tumor proliferation and metastasis [37, 38]. Therefore, by inhibiting the activity of PI3K/AKT, tumor cells can undergo apoptosis, thereby inhibiting their proliferation and metastasis. This method can be used to treat acute lymphoblastic leukemia. In this study, the expression of CCL3, its receptor CCR5, and PI3K were also positively correlated. Hence, there may be a cascade activation network relationship between chemokines and PI3K/AKT in the process of tumor invasion and metastasis. These factors affect each other, and lead to tumor proliferation and invasion. Therefore, in the treatment of tumors, the activation and release of other factors can be controlled to inhibit tumor proliferation through the administration of effective drugs that can interfere with any one of these factors.

In 1969, Rygaard and Povlsen first succeeded in transplanting excised specimens of human cancer tissue into nude mice. Since then, animal models of transplanted tumors have been widely used in the study of tumor growth and metastasis. Methods commonly used to establish colorectal cancer xenograft animal models include cell and tissue transplantation. Athymic nude mice or severely combined immunodeficient (SCID) mice are generally used to reduce the impact of rejection and the killing effect of immune cells on tumor cells during modeling [39]. The xenotransplantation model has a high tumor formation rate, short cycle, and low rates of immune rejection. It is mainly used for research on human tumors to investigate the treatment, invasion, and metastasis mechanisms, as well as drug sensitivity. The model retains the original morphology and biological characteristics of tumor cells and can dynamically observe tumor formation. Moreover, it exhibits good repeatability and is convenient for monitoring tumor progression and detecting related cytokines. Furthermore, it is effective in screening drug safety and evaluating the effect of pharmacological interventions. However, it is difficult to replicate the occurrence of metastases using this model. Human-derived cell lines are widely used in HCT116 and HT29 cell lines [40]. The subcutaneous tumor model selected in this experiment is very helpful for observing the growth state of the tumor.

Tanabe [41] used the mouse-derived colon cancer cell line colon26 to establish a cecal xenograft model in wild-type BALB/c mice. Injection of the CCR5 inhibitor maraviroc into mice-inhibited tumor proliferation and reduced the expression of CCL3, CCL4, and CCL5. Da [15] studied the transplanted tumor model of oral squamous cell carcinoma. The results showed that knockout CCL3−/− mice and CCR5−/− wild-type C57BL/6 mice exhibited slower tumor proliferation, and the difference was statistically significant. These findings are consistent with the results of this experiment. However, in the present study, we used BALB/c nude mice, which relatively reduced the impact of the immune system. At the same time, we used a human cell line to confirm the expression of CCL3. In a previous study, SCID mice were subcutaneously injected with HT29 cells (10 × 10^6^) [42]. After 22 days of feeding, 100% of the experimental mice had developed lung metastasis. Nevertheless, in our experiments, there was no obvious lung metastasis found.

Ki67 protein (also termed as mKi67) is a marker that reflects cell proliferation [43]. During mitosis, the Ki67 protein is relocated to the surface of the chromosome; during the intercellular phase, the Ki67 antigen can only be detected in the nucleus. The level of Ki67 protein increases significantly when the cell progresses to the *S* phase of its cycle [44], and its expression level is considered a marker for the proliferation of breast cancer cells [45]. In clinical practice [46], Ki67 is routinely used clinically to assess whether patients with colorectal cancer require further adjuvant chemotherapy. Studies have confirmed that the Ki67 index is a surrogate indicator for predicting the efficacy of neoadjuvant chemotherapy. In this study, we detected Ki67 in subcutaneous xenograft tumors of colon cancer to further verify that enhanced or weakened secretion of CCL3 is positively correlated with tumor proliferation [47].

The limitations of this study are as follows. Firstly, this investigation did not include control study of wild-type BFT because the extraction of wild-type BFT is challenging. Secondly, in the clinical pathological correlation study, we did not perform a survival and prognosis correlation analysis using the selected case data. Finally, the sample size of the animal experiments needs to be expanded, and in-depth research on the mechanism of BFT-1 and colon cancer cells is warranted.

## 3. Materials and Methods

### 3.1. Inclusion and Exclusion Criteria

The criteria were as follows: (1) all patients were clearly diagnosed with colorectal cancer after pathological examination, and confirmed to undergo radical surgery for colorectal cancer; (2) patients aged 40–75 years; (3) no edematous diseases prior to the operation, such as pleural effusion and ascites effusion, no cachexia, no intestinal obstruction, no serious cardiopulmonary dysfunction, and no wasting disease; (4) no radiotherapy or chemotherapy performed prior to the operation; (5) no significant metastasis of cancer cells to important organs before operation; (6) no obvious abnormality in the liver and kidney function; (7) no congenital metabolic disease; (8) ability of patients to stand and walk at the time of admission to the hospital; (9) no usage of antibiotics 1 month prior to the operation; and (10) no infectious disease and no inflammatory disease (cholecystitis, gastrointestinal inflammatory disease, viral hepatitis, nephritis, autoimmune system disease, rheumatoid arthritis, and ankylosing spondylitis) prior to the operation.

### 3.2. Cytokine Array Analysis

#### 3.2.1. Human Specimens

This experiment was approved by the Ethics Committee of Ningxia Medical University General Hospital, Yinchuan, China (approval number: 2017-200), and prior to the selection of materials, patients and their families provided written informed consent. The researchers obtained 16 samples from four patients with colorectal cancer. The samples were surgically resected in the General Hospital of Ningxia Medical University from September 2019 to March 2020: normal (*n* = 3); paracancer (*n* = 3); adenomas (*n* = 3); cancer (*n* = 4); and metastatic lymph nodes (*n* = 3). Normal samples and paracancerous tissues were obtained from the intestinal tissue >5 cm and 3–5 cm away from the cancer, respectively. The adenomatous tissue was taken from the adenomatous polyp tissue in the intestinal tract (except for the tumor), and pathological examination revealed adenoma. The metastatic lymph node tissue was taken from the regional metastatic lymph node tissue confirmed by the frozen section during the operation. The cancer tissue was taken from the whole layer tissue block of colorectal cancer diagnosed by preoperative pathology. All samples were collected within 30 min after surgical removal of the specimens. Fresh samples were washed with phosphate-buffered saline (PBS) solution, immediately frozen in liquid nitrogen, and transferred to −80°C.

#### 3.2.2. Cytokine Array Analysis

Proteins of the surgical specimens were extracted through cutting the tissues into small pieces, homogenizing and lysing them using homogenizer and cell lysis buffer (Sigma, USA). And the concentration was valued by BCA assay kit (KeyGEN Biotech, China). After blocking and incubation of the certain anti-cytokine chip (RayBio, China), the proteins were incubated with the chip at 4°C overnight. Following that, the chip was washed, blocked, and then incubated with biotin-labeled antibody. Finally, after washing, the proteins were visualized using HRP-Streptavidin (Sigma, USA) and scanned with a chemiluminescence imaging analysis system (ImageQuant LAS4000). The AAH-CHE-1-8 data analysis software was used for data analysis. Differentially expressed genes were obtained and subjected to the Kyoto Encyclopedia of Genes and Genomes enrichment analysis to determine the significant biological regulatory pathways involved in the progression of CRC. Fisher's exact test and R language were used in this experiment for the enrichment analysis. The node/path data was sorted in descending order according to the value of the count. The gene order of difference on a certain node/path ≥5 was the criterion for the selection of factors and pathways with significant differences.

### 3.3. Cell Lines, Cell Culture, and Lentivirus Vectors Infection

CRC cell lines (SW620, HT29, and HCT116) and normal colon cell line (NCM460) were purchased from ATCC (American Type Culture Collection, VA, USA). Cells were collected and cultivated at 37^o^C in an incubator with 5% CO_2_ in different medium (SW620: Leibovitz's L-15 medium, HT29 and HCT116: McCoy's 5A medium, and NCM460: RPMI-1640 medium) supplemented with 10% fetal bovine serum (FBS), 100 U/ml penicillin, and 100 *μ*g/ml streptomycin (Gibco, Invitrogen, USA). Lentivirus vectors carrying shRNA-CCL3 or CCL3 OE plasmids were constructed, and then they were infected to the CRC cells at certain MOI to downregulate or upregulate the expression of CCL3 in CRC cells.

### 3.4. Western Blotting

The cells were taken from the incubator to remove the culture medium and washed twice with precooled PBS. Proteins were harvested using whole cell lysis assay (KeyGEN Biotech, China) according to the manufacturer's instructions. After valuing the concentration and equaled the quantity of loading samples, the proteins of different groups were separated by SDS-PAGE and subsequently transferred onto PVDF membranes (Millipore, MA, USA). Afterwards, the membranes were blocked with 5% nonfat milk in TBST at room temperature for 1 h, followed by incubation with antibodies against targeting protein overnight at 4°C. The primary antibodies including anti-CCR5, anti-TRAF6, anti-NF-kB, and anti-PI3K were purchased from Abcam (Cambridge Science Park, UK), and used as the following concentration: anti-CCR5: 1 : 1000; anti-TRAF6:1 : 2000; anti-NF-kB:1 : 500; anti-PI3K:1 : 250; and anti-*β*-Actin:1 : 5000. Following being washed with TBST buffer, the membrane was stripped with appropriate HRP-conjugated secondary antibodies (Abcam, CA, USA) for 1 h at room temperature, followed by visualized using the enhanced Western Bright ECL reagents (Cell Signaling Technology, USA). Eventually, bands were imaged and analyzed by a chemiluminescence detection system (Bio-Rad, USA). The experiments were repeated at least three times to ensure reproducibility.

### 3.5. Enzyme-Linked Immunosorbent Assay (ELISA) Human MIP-1*α*/CCL3 ELISA

ELISA Kit (Boster technology, China) was used to detect the secretion of CCL-3 from normal colon epithelial and CRC cells. According to the manufacturer's protocol, a standard curve for duplicate measurements was constructed. Then, at certain time points, the cells culture media were centrifuged at 2,000× g for 10 minutes to remove debris and supernatants were collected and diluted by the sample dilution provided. Add 100 *μ*L of samples or standard to appropriate wells. Seal the plate and incubate for 90 minutes at 37°C on a plate shaker set to 400 rpm. Remove the liquids and add 100 *μ*L of the anti-CCL3 antibody to each well. Seal the plate and incubate for 60 minutes at 37°C on a plate shaker set to 400 rpm. Wash each well with 3 × 350 *μ*L wash buffer and after the last wash invert the plate and blot it against clean paper towels to remove excess liquid. Add 100ul of the prepared ABC work solution. Seal the plate and incubate for 30 min. Wash each well with 5 × 350 *μ*L wash buffer and after the last wash invert the plate and blot it against clean paper towels to remove excess liquid. Add 100 *μ*L of TMB substrate to each well and incubate for 20 minutes in the dark on a plate shaker set to 400 rpm. Add 100 *μ*L of stop solution to each well. Shake the plate on a plate shaker for 1 minute to mix. Record the OD at 450 nm using an ELISA reader (Bio-Rad Laboratories, Richmond, CA, USA).

### 3.6. Cell Counting Kit-8 (CCK8) Experiment

The proliferations of HT29 and HCT116 cells with the impression of CCL3 were determined by Cell Counting Kit-8 (CCK-8) assay according to the manufacturer's instructions using Cell CountingKit-8 (Dojinodo, Shanghai, China). In brief, cells with inhibition or overexpression of CCL3 were plated in 96-well microplates. Once the cells were stickled to the bottom of plates, the proliferation was detected (0 h), and then, it was also detected at 12 h, 24 h, 36 h, 48 h, and 72 h. For detection, the CCK-8 solution (10 *μ*l) was added to each well and incubated for additional 4 h. Absorbance at 450 nm was measured using an ELISA reader (Bio-Rad Laboratories, Richmond, CA, USA).

### 3.7. Transwell migration and Invasion Experiment

The migration and invasion of HT29 and HCT116 cells with the impression of CCL3 were determined by transwell migration and invasion assays. For transwell migration assays, the cells were cultured without FBS for 6 h, and then equal quantity of cells in different groups were harvested with 200 *μ*L FBS free culturing medium and seeded into the 8.0 *μ*m pore polycarbonate membrane inserts (Corning, USA). Meanwhile, medium (500 *μ*l) containing 30% fetal bovine serum was added to the lower chamber of the 24-well plate. The cells were conventionally cultured for 48 h. The cell culture medium was aspirated, and the cells were washed twice with PBS. The cells in the upper surface were removed using a wet cotton ball and the cells remained were stained with 0.1% crystal violet for 20 min. After being gently washed twice with PBS to remove excess staining, the cells were pictured and counted. For transwell invasion assays, the upper 8.0 *μ*m pore polycarbonate membrane inserts (Corning, USA) of the transwell were pre-coated with 50 mg/l Matrigel (BD, USA) diluent (1 : 8). And the subsequent procedures were the same with those in the transwell migration assays.

### 3.8. Cell Scratch Detection

The density of different groups of cells was adjusted to 6 × 10^5^ cells/mL; the cells were seeded into 6-well plates and cultured until the cell density reached approximately 100%. The cell layers were scratched with a sterile 10 *μ*l pipette tip *p* and washed twice with PBS. With 0 h and 24 h incubation, 3 fields were visualized to assess migration. The scratch area was calculated using the ImageJ software (National Institutes of Health, Bethesda, MD, USA), and one-way analysis of variance was employed to analyze the input data.

### 3.9. Immunohistochemistry (IHC) Assays

#### 3.9.1. Collection of Human Specimens for IHC

According to inclusion and exclusion criteria, tissues including cancer, para-cancer, and normal epithelial colorectal tissue were collected from 50 patients diagnosed with CRC to perform immunohistochemistry assays. Meanwhile, the clinical data of 50 patients were also collected. Among them, 26 and 24 patients were males and females, respectively; 19 and 31 patients were aged ≤60 years and >60 years, respectively. Moreover, the cancer of 22 and 28 patients located in rectum and colon, respectively; 14, 17, and 19 patients had TNM stage I, II, and III disease, respectively. The degree of differentiation was as follows: high (seven cases), moderate (30 cases), and poor (13 cases). There were 16 and 34 cases with and without vascular invasion, as well as 22 and 28 cases with and without nerve invasion, respectively.

#### 3.9.2. Immunohistochemistry Staining

The surgically resected tumor samples were fixed with 10% neutral formalin and subsequently embedded in paraffin. A 4-*μ*m thickness of sections were deparaffinized and rehydrated through graded alcohol solution, and then boiled in 10 mm sodium citrate pH 6.0 for 15 min in an autoclave and cooled down to room temperature (RT) for a purpose of antigen retrieval. Then, under RT conditions, it was treated with 3% hydrogen peroxide for 20 minutes to eliminate endogenous peroxidase activity. The sections were incubated with blocking buffer (5% goat serum in PBS) for 2 h at RT to block the nonspecific binding. Tissue sections were then incubated with primary antibodies including rabbit anti-human CCL3 antibody (1 : 50, ab32609, Abcam, Cambridge Science Park, UK), goat anti-human CCR5 antibody (1 : 300, ab65850, Abcam, Cambridge Science Park, UK) overnight at 4 °C. Paralleled sections were incubated with rabbit and mouse IgG to become isotype controls. After washing with PBS, horseradish peroxidase (HRP)-conjugated goat anti-rabbit IgG antibody (zb2301, ZSGB-BIO, Beijing, China) or peroxidase-conjugated goat anti-mouse IgG antibody (zb2307, ZSGB-BIO, Beijing, China) were used as secondary antibodies and incubated for 2 h at RT. After washing with PBS, the sections were incubated with 3′-diaminobenzidine (DAB) peroxidase substrate and counterstaining with hematoxylin. The images of stained sections were captured with the high-powered upright microscope (Leica DM3000). Gray-level density mean and numbers of positive-CCL3 and CCR5 cells were analyzed by Image Pro Plus 6 (IPP6).

#### 3.9.3. Data Analysis of Immunohistochemistry Assays

The IHC stained sections were then blindly evaluated by three independent pathologists. The appearance of yellow-brown particles in the cytoplasm of the cells was indicative of positivity for CCL3 and CCR5. This positivity was graded according to the intensity of cytoplasmic staining: 0 (negative), 1 (weak positive), 2 (moderate positive), and 3 (strong positive). The classification according to the scope of staining was as follows: 0 points (<5%), 1 point (5–25%), 2 points (26–50%), 3 points (51–75%), and 4 points (>75%). The staining intensity was multiplied by the staining range to obtain the immunohistochemical score: no expression (0), low expression (0–4), moderate expression (5–8), and high expression (9–12). Moreover, the correlation between the IHC data and clinal features of the patients were analyzed using SPSS 23.0.

### 3.10. Subcutaneous Tumorigenicity in Nude Mice

#### 3.10.1. Animals

Female BALB/c nude mice (*n* = 36) (specific-pathogen-free (SPF) grade, age: 4 to 6 weeks; weight: 16–18 g) were purchased from Beijing Weitong Lihua Experimental Animal Center (Beijing, China). The mice were raised in the SPF barrier animal laboratory of the Experimental Animal Center of Ningxia Medical University. The feed (SPF-level AIN-93G purified) was purchased from Beijing Keaoli Feed Co., Ltd. (Beijing, China). The mouse feed was changed once every 5 days. The water was filtered and sterilized by high temperature and high pressure. The experimental conditions of daily animal care were based on the standards for laboratory animal environment and facilities of the ministry of health of the People's Republic of China. All animal experiments were approved by the Laboratory Animal Management Committee of Ningxia Medical University and conducted in accordance with the National Institutes of Health Animal Ethical Use Guidelines. The experiments were reviewed by the Ethics Committee of Ningxia Medical University.

#### 3.10.2. Subcutaneous Tumorigenicity Assays

The 36 nude mice were divided into two groups, and then, 3 subgroups named the control, empty vector (NC), and interference/overexpression groups(shRNA/OE). 1 × 10^7^ differentially treated HT29 or HCT116 cells including control-HT29, NC-HT29, shRNA CCL3-HT29, control-HCT116, NC-HCT116, and OE CCL3-HCT116 in 200 *μ*l normal saline. The maximum diameter of the tumor was measured once every 5 days and the curve of tumor growth was drawn. When the maximum diameter of the tumor reached 1.5 to 2 cm, the nude mice were sacrificed, immunohistochemical methods were used to detect the expression of Ki67 in tumor specimens and determine the effect of CCL3 on tumor proliferation.

### 3.11. Statistical Analysis

Data were expressed as the mean ± standard error. One-way analysis of variance, *t*-test, and nonparametric test were used to conduct group comparisons. Categorical variables were compared using chi-squared test. SPSS 22.0 and GraphPad Prism 5.0 were used. *P* < 0.05 was considered to be indicated as statistically significant difference.

## 4. Results

### 4.1. Protein Array for Chemokines

Based on the analysis of the standardized optical density values obtained from the membrane array, it is suggested that CCL3 are highly expressed in cancer tissues and metastatic cancer tissues; the difference was statistically significant (*P* < 0.05), as shown in Figure 1 and Table 1. In Figure 1, the red box indicates the optical density expression map of the membrane array of the chemokines CCL3, CCL4, and IL8.

### 4.2. Colorectal Adenoma-Cancer Sequence in Different Group Target Chemokine Screening Optical Density Data Statistical Table

The difference in the standardized optical density between samples, as the criterion for screening differentially expressed proteins, was statistically significant (*P* < 0.05). The antibody array chemokine enrichment analysis chart shows that the chemokines CCL3, CCL4, and IL8 were highly expressed in colorectal cancer tissues and metastatic lymph nodes; however, they were downregulated in the normal, adjacent, and adenoma groups. The difference was statistically significant (*P* < 0.05), as shown in Figure 2. Because CCL4 did not achieve the expected results in the subsequent cell verification process, the high expression of IL8 factor in colorectal cancer and a variety of cancers has been confirmed. Thus, we finally selected CCL3 as the target factor. In Figure 2, the red and green parts indicate that the gene was upregulated and downregulated, respectively. The red circle indicates the chemokine CCL3.

### 4.3. Verification of Factor Expression at the Tissue Level Using Western Blotting

Compared with normal tissues, CCL3 was highly expressed in cancer tissues, while CCR5, NF-*κ*B, TRAF6, and PI3K were highly expressed in cancer tissues and metastatic lymph nodes. The difference was statistically significant (*P* < 0.05). We compared the protein expression levels of cancer and paracancerous tissues. The expression level of TRAF6 increased in paracancerous tissue, and the difference was statistically significant (*P* < 0.05). However, western blotting showed that the expression levels of these factors in cancer tissue and metastatic lymph node tissue were not significantly different (*P* > 0.05), as shown in Figure 3.

### 4.4. Expression of Chemokine CCL3 in Colorectal Cancer Tissues, Paracancerous Tissue, and Normal Tissues Using Immunohistochemistry

CCL3 is mainly expressed in the cytoplasm and outside the cell. It is highly expressed in cancer tissues (brown or brownish yellow) as well as in paracancerous tissues and normal tissues. The expression gradually decreases from paracancerous to cancerous tissues. All extracellular lymphocytes express CCL3. According to the analysis of immunohistochemical scores, the expression of CCL3 in normal and paracancerous colorectal cancer tissues gradually increased, and the difference between the groups was significant (*P* < 0.05), as shown in Figure 4.

### 4.5. Expression of Chemokine CCR5 in Colorectal Cancer Tissues, Paracancerous Tissues, and Normal Tissues through Immunohistochemistry

CCR5 is mainly expressed in the cytoplasm. It is highly expressed in cancerous tissues (brown or brownish yellow) as well as in paracancerous tissues and normal tissues. Its expression gradually decreases from paracancerous to cancerous tissues. In paracancerous and normal tissues, CCL3 is expressed on lymphocytes outside colonic epithelial cells. According to the analysis of immunohistochemical scores, the expression of CCR5 in normal and paracancerous colorectal cancer tissues gradually increased, and the difference between the groups was significant (*P* < 0.05), as shown in Figure 5.

### 4.6. Correlation Analysis between the Expression of CCL3 and CCR5 in Human Colorectal Cancer Tissues and Clinical Data

As shown in Table 2, according to the immunohistochemical score, further statistical analysis showed that the expression level of CCL3 was correlated with TNM staging (*P* < 0.05). Subsequently, after further segmentation testing on TNM staging, it was found that the expression of CCL3 was significantly different among patients with stage 1 and 3 colorectal cancer (*P* < 0.05); however, there was no correlation with other clinical indicators (*P* > 0.05). ^*∗*^The split test within the group was further performed after conducting the chi-squared test.

As shown in Table 3, further statistical analysis based on the immunohistochemical score revealed that the expression level of CCR5 was correlated with TNM staging (*P* < 0.005) and nerve invasion (*P* < 0.05); however, there was no correlation with other clinical indicators (*P* > 0.05). ^∗^ indicates that the split test within the group was further performed after conducting the chi-squared test.

### 4.7. CCL3-HT29 Interference and CCL3-HCT116 Overexpression Cell Proliferation

The tumor proliferative ability of CCL3 was weakened after RNA interference; while the proliferative ability of HCT116 cells was enhanced after overexpression of CCL3. The difference was statistically significant (*P* < 0.05). The differences in proliferative ability were all manifested 12 h following resuscitation of colon cancer cell lines, as shown in Figure 6.

### 4.8. Transwell Cell Migration Experiment

The results of the Transwell cell invasion experiment suggested that the invasive ability of HT29 cells was weakened after RNA interference with CCL3. Following overexpression of CCL3, the migratory ability of HCT116 cells was enhanced, and the difference was statistically significant (*P* < 0.05), as shown in Figure 7.

### 4.9. Pathway Gene Expression by Western Blotting

#### 4.9.1. Expression of Pathway-Related Genes in Colon Cancer HT29 Cells after CCL3 Interference

After CCL3 interference, the expression of CCR5, NF-*κ*B, TRAF6, PI3K, and the normal decreased, and the difference was statistically significant (*P* < 0.05). However, the difference in expression between the control group and NC group was not statistically significant (*P* > 0.05), as shown in Figure 8.

#### 4.9.2. Expression of Pathway-Related Genes after CCL3 Overexpression in Colon Cancer HCT116 Cells

After overexpression of CCL3, the levels of CCR5, NF-*κ*B, TRAF6, and PI3K were increased; the difference was statistically significant (*P* < 0.05), as shown in Figure 9.

### 4.10. Effects of Interference and CCL3-Overexpressing Colon Cancer Cell Lines on Tumor Formation in Nude Mice

#### 4.10.1. CCL3 Interference in HT29 Cells

After CCL3 interference, the tumor proliferation in HT29 cells was retarded. Compared with the control group, the tumor diameter decreased significantly (*P* < 0.05). The control and empty vector groups did not show statistically significant differences in tumor proliferation (*P* > 0.05), as shown in Figure 10.

#### 4.10.2. CCL3 Overexpression in HCT116 Cells

Overexpression of CCL3 in HCT116 cells accelerated tumor proliferation, and the difference in tumor diameter compared with the control group was statistically significant (*P* < 0.05). Moreover, the difference in tumor proliferation between the control and empty vector groups was not statistically significant (*P* > 0.05), as shown in Figure 11.

### 4.11. Immunohistochemical Detection of Ki67 in Nude Mice

#### 4.11.1. Effects of CCL3 Interference on Ki67 in Stably Transfected Cells

After CCL3 RNA interference in colon cancer HT29 cells, the expression of Ki67 was decreased, and the tumor proliferative ability of cells was weakened. The difference was statistically significant (*P* < 0.05). The difference in tumor proliferation between the control and empty vector groups was not statistically significant (*P* > 0.05), as shown in Figure 12.

#### 4.11.2. Immunohistochemical Testing of Ki67 in CCL3-Overexpressing Stably Transgenic Cells

Following overexpression of CCL3 in colon cancer HCT116 cells, the expression of Ki67 was increased, and the tumor proliferative ability of cells was enhanced. The difference was statistically significant (*P* < 0.05). The difference in tumor proliferation between the control and empty vector groups was not statistically significant (*P* > 0.05), as shown in Figure 13.

## 5. Conclusions

In this study, the cell, tissue, and animal experiments were conducted to prove that CCL3 is highly expressed in colorectal cancer. The experimental results confirmed that CCL3 can promote the proliferation of cancer cells, and its expression is closely related to TRAF6/NF-*κ*Bmolecular pathway. CCL3 and CCR5 were expressed in paracancerous tissues, colorectal cancer tissues, and metastatic carcinoma, and the degree of expression was correlated with clinical stage and nerve invasion. The expression of chemokine CCL3 and receptor CCR5 is positively correlated with the expression of TRAF6 and NF-*κ*B and can promote the proliferation, invasion, and migration of colorectal cancer through TRAF6 and NF-*κ*B pathway.

## Figures and Tables

**Figure 1:** Results of the adenoma cancer sequence antibody membrane array: (a) normal tissue; (b) paracancerous tissue; (c) cancer tissue; (d) metastatic tissue.

**Figure 2:** Differential chemokine enrichment analysis between different groups of the adenoma cancer sequence by protein array analysis: (a) normal and cancerous tissue; (b) normal and metastatic lymph node tissue; (c) cancer and adjacent tissue; and (d) cancer and adenoma tissue.

**Figure 3:** Western blotting to verify the expression levels of CCL3, CCR5, and the TRAF6/NF-*κ*B pathway-related factors in colorectal cancer tissues: (a) the expression level of CCL3 in different colorectal cancer tissues; (b) a graph of the expression level of CCR5 in different colorectal cancer tissues; (c) changes in the expression level of NF-*κ*B in different colorectal cancer tissues; (d) a graph of changes in the expression of TRAF6 in different colorectal cancer tissues; and (e) changes in the expression level of PI3K in different colorectal cancer tissues.

**Figure 4:** Immunohistochemical detection of CCL3 expression in colorectal cancer tissues, paracancerous tissues, and normal tissues: (a) CCL3 expression in colorectal cancer tissue (×200); (b) CCL3 expression in colorectal cancer tissue (×400); (c) the expression of CCL3 in colorectal paracancerous tissues (×200); (d) the expression of CCL3 in colorectal paracancerous tissues (×400); (e) CCL3 expression in normal colorectal tissues (×200); (f) CCL3 expression in normal colorectal tissues (×400); and (g) scatter plot comparing the immunohistochemical scores of colorectal cancer, paracancerous tissues, and normal tissues.

**Figure 5:** Immunohistochemical detection of CCR5 expression in colorectal cancer tissues, paracancerous tissues, and normal tissues: (a) CCR5 expression in colorectal cancer tissue (×200); (b) CCR5 expression in colorectal cancer tissue (×400); (c) CCR5 expression in colorectal paracancerous tissues (×200); (d) CCR5 expression in colorectal paracancerous tissues (×400); (e) CCL3 expression in normal colorectal tissues (×200); (f) CCR5 expression in normal colorectal tissues (×400); (g) scatter plot comparing the immunohistochemical scores of colorectal cancer, paracancerous tissues, and normal tissues.

**Figure 6:** CCL3 interference and overexpression in the CCK8 proliferation experiment: (a) CON: Colon cancer HT29 cells, NC: HT29 cells stably transfected with empty vector, ShRNA: CCL3-HT29 cells stably transfected with interference shRNA for CCL3; (b) CON: Colon cancer HCT116 cells, NC: HCT116 cells stably transfected with empty vector, OE: CCL3-HCT116 cells stably transfected for overexpression of CCL3.

**Figure 7:** Results of the transwell invasion experiment for CCL3 interference and overexpression: (a) HT29 cell invasion for 12 h; (b) graph of the statistical analysis of HT29 cell invasion; (c) HCT116 cell invasion for 12 h; and (d) graph of the statistical analysis of HCT116 cell invasion.

**Figure 8:** The expression levels of related factors in colon cancer HT29 cells after CCL3 RNA interference: (a) western blotting results for CCR5 and TRAF6/NF-*κ*B pathway-related factors; (b) graph of the statistical analysis for the expression of factors.

**Figure 9:** The expression levels of related factors after CCL3 RNA overexpression in colon cancer HCT116 cells: (a) western blotting results are CCR5 and TRAF6/NF-*κ*B pathway-related factors in HCT116 cells; (b) chart of the statistical analysis for the differential expression of each factor.

**Figure 10:** Tumor formation in nude mice after CCL3 interference in HT29 cells: (a) schematic diagram of tumor formation in nude mice with HT29 cells and their stable transgenic strains; (b) statistical analysis of the tumor diameter in each group; and (c) tumor growth curve of nude mice, Con: control group, NC: empty vector group, and ShRNA: CCL3 interference group.

**Figure 11:** Tumor formation in nude mice after CCL3 overexpression in HCT116 cells: (a) a schematic diagram of tumor formation in nude mice with HCT116 cells and their stable transgenic strains; (b) statistical analysis of the tumor diameter in each group; and (c) tumor growth curve. Con: control group, NC: empty vector group, and OE: CCL3 overexpression group.

**Figure 12:** Immunohistochemical map of tumorigenesis Ki67 in CCL3 interference stable transgenic HT29 cells: (a) immunohistochemical images of the three groups for the detection of tumor tissue Ki67 in the HT29 subcutaneous tumor formation experiment; (b) H-score statistical analysis of the immunohistochemistry results.

**Figure 13:** Immunohistochemical map of tumorigenesis Ki67 in CCL3 overexpression stable transgenic HCT116 cells: (a) immunohistochemical images of the three groups for the detection of tumor tissue Ki67 in the HCT116 subcutaneous tumor formation experiment; (b) H-score statistical analysis of the immunohistochemistry results.

**Table 1:** Dot matrix for chemokine antibody identification.

	A	B	C	D	E	F	G	H	I	J	K	L

1	Pos	Pos	NEG	NEG	BLC (CXCL13)	CCL28(MEC)	CK beta8-1 (CCL23)	CTACK (CCL27)	CXCL16	ENA-78(CXCL5)	Eotaxin-1 (CCL11)	Eotaxin-2(CCL24)
2	Eotaxin-3(CCL26)	Fractalkine (CX3CL1)	GCP-2 (CXCL6)	GRO a/b/g/	GRO alpha (CXCL1)	HCC-4(CCL16)	I-309(TCA-3/CCL1)	TAC (CXCL11)	IL8(CXCL18)	IP-10(CXCL10)	Lymphotactin	MCP-1(CCL2)
3	MCP-2(CCL8)	MCP-3 (CCL7)	MCP-4(CCL13)	MDC (CCL22)	MIG(CXCL9)	MIP-1 alpha(CCL3)	MIP-1beta (CCL4)	MIP-1 delta (CCL15)	MIP-3 alpha (CCL20)	MIP-3 beta	MPIF-1(CCL23)	NAP2(CXCl7)
4	PARC(CCL18)	RANTES (CCL5)	SDF-1 alpha	SDF-1 beta	TARC(CCL17)	BLANK	BLANK	BLANK	BLANK	BLANK	BLANK	Pos

**Table 2:** Correlation analysis of CCL3 expression and clinical data in human colorectal cancer tissue.

Group	*n*	CCL3 expression				*χ* ^2^	*P*
		High	Moderate	Low	Loss		

Gender							
Male	26	5	14	6	1	3.559	0.313
Female	24	3	16	2	3		
Age							
≤60 years	19	3	14	1	1	5.949	0.114
>60 years	31	5	15	8	3		
Tumor site							
Rectum	22	2	16	4	0	5.785	0.123
Colon	28	6	13	5	4		
TNM stage							
I	14	1	4	8	1	18.442	0.005^*∗*^
II	17	4	9	3	1		
III	19	4	13	0	2		
Differentiation (grade)							
Well	7	0	4	2	1	9.95	0.127
Moderate	30	6	18	4	2		
Poor	13	7	4	1	1		
Lymph-vascular space invasion							
Present	16	3	9	3	1	0.73	0.886
Absent	34	5	20	6	3		
Perineural invasion							
Present	22	3	16	3	0	5.165	0.16
Absent	28	5	13	6	4		

**Table 3:** Correlation analysis of CCR5 expression and clinical data in human colorectal cancer tissue.

Group	*n*	CCL5 expression				*χ* ^2^	*P*
		High	Moderate	Low	Loss		
Gender							
Male	26	10	12	4	0	2.11	0.55
Female	24	10	8	4	2		
Age							
≤60 years	19	7	7	3	2	0.076	0.962
>60 years	31	12	13	6	0		
Tumor site							
Rectum	22	10	9	3	0	2.314	0.51
Colon	28	11	11	4	2		
TNM stage							
1	14	4	4	6	0	19.994	0.003^*∗*^
2	17	7	7	1	2		
3	19	11	8	0	0		
Differentiation (grade)							
Well	7	2	1	2	1	7.074	0.314
Moderate	30	14	11	3	1		
Poor	13	5	8	2	0		
Lymph-vascular space invasion							
Present	16	5	9	3	0	5.811	0.121
Absent	34	16	11	1	2		
Perineural invasion							
Present	22	8	12	1	0	8.689	0.034
Absent	28	13	7	7	2		

## Data Availability

At present, the datasets used and analyzed during the current study are available from the corresponding authors on reasonable request.

## Abbreviations

CCL3: Chemokine C-C motif chemokine ligand 3
TLR/NF-*κ*B: The toll-like receptors/nuclear factor-*κ*b
TNF: Tumor necrosis factor
CCR5: C-C motif chemokine receptor 5
CCR1: C-C motif chemokine receptor 1
HIV-1: Human immunodeficiency virus type 1
PKC: Protein kinase C
NF-*κ*B: Nuclear factor-*κ*B
PI3K: The phosphatidylinositol-3-kinase
TRAF6: TNF receptor-associated factor 6
AP-1: Activator protein-1
CCK8: Cell counting kit-8
IHC: Immunohistochemistry
HRP: Horseradish peroxidase
DAB: Diaminobenzidine
IPP6: Image Pro Plus 6
CCL4: Chemokine C-C motif chemokine ligand 4
IL8: Interleukin 8
TLR: The toll-like receptors
MMP: Matrix metalloproteinases
SCID: Severely combined immunodeficient
CCL5: Chemokine C-C motif chemokine ligand 5.
